# Study on the Clinical Characteristics and Treatment of Obstetric Hypertension with Sequence Pattern Mining Algorithm

**DOI:** 10.1155/2021/1072446

**Published:** 2021-09-27

**Authors:** Jiawei Li

**Affiliations:** Guangdong Women's and Children's Hospital, Guangdong 510000, Guangzho, China

## Abstract

Aiming at the difficulty in setting the support threshold for sequential pattern mining algorithms and improving the effectiveness of the support threshold setting without the guidance of domain experts' experience, an improved SPADE (sequential pattern discovery using equivalence classes) algorithm is proposed. By analyzing the relationship between the number of frequent sequences and the support threshold, the support threshold is dynamically selected. Using the electronic medical record data from a medical centre, the time-series relationship of the drugs taken by hypertension patients was extracted as the drug sequence dataset. By determining the optimal support threshold of the dataset, the frequent sequence set is mined, and the sequence rules are generated from the obtained regular sequences to visualize the sequence rules. The sequence rules of medication for hypertensive patients were combined with the patients' physical indicators for the recommendation. For patients with obstetric hypertension, a combination of nifedipine and captopril is recommended. Through the comparison of the observation group and control group, we study the curative effect of various drugs. The results showed that the total effective rate of the observation group was about 96.6%; compared with the control group, the result indicated that the difference was significant (*P* < 0.05). The comparison of blood pressure levels between the two groups after treatment also showed that the results of the observation group were ideal (*P* < 0.05). In addition, the incidence of postpartum haemorrhage and perinatal complications in the observation group was also significantly reduced (*P* < 0.05). Therefore, the combination of medication for pregnancy hypertension syndrome can effectively improve the treatment effect of the disease and reduce the rate of postpartum haemorrhage and the incidence of perinatal complications.

## 1. Introduction

Pregnancy hypertension syndrome is a widespread type of clinical complication, which can occur in the prenatal, delivery, and postpartum time. The disease can lead to clinical symptoms such as elevated blood pressure, oedema, and proteinuria. Patients with severe disease may even have adverse consequences such as coma, heart failure, and kidney failure, which poses a severe threat to the pregnancy outcome of pregnant women. At present, the pathogenesis of pregnancy hypertension is not completely clear, and the clinical treatment of pregnancy hypertension syndrome is mainly composed of sedation, spasmolysis, and hypotension. Relevant studies have found that the use of antihypertensive drugs in patients with pregnancy hypertension syndrome is helpful to reduce the level of blood pressure of patients, improve the clinical treatment effect, and reduce the incidence of various complications.

Sequential pattern mining was first proposed by Algrawal et al. and Apriori algorithm and multilevel iterative algorithm were proposed to study customer purchase behavior in retail industry. SPADE algorithm is a sequential pattern mining algorithm proposed by Zaki and others. Because of the shortcomings of the GSP algorithm that needs to scan the database multiple times, the SPADE algorithm uses a vertical storage structure based on lattice theory and the idea of equivalent classes to reduce the number of database scans to 3. It reduces the time complexity.

At present, research on reducing pregnancy-induced hypertension in patients is developing. Yata et al. applied laser speckled flow imaging (LSFG) and enhanced depth imaging optical coherence tomography (EDI-OCT) techniques to observe the changes of choroid blood flow (CBF), choroid pulse waveform, and central choroid thickness (CCT) in patients with pregnancy hypertension syndrome (PIH) before and after treatment [1]. He et al. discussed the efficacy and safety of magnesium sulfate which was combined with low-dose aspirin in the treatment of PIH [2]. Gao et al. addressed the application of Doppler ultrasound in Omaha system nursing intervention (NI) to monitor the changes of important blood vessel hemodynamic indexes of pregnant women with PIH during pregnancy [3]. Vani et al. studied the incidence of pregnancy hypertension syndrome and related risk factors [4].

Sequential pattern mining algorithms are constantly developing. Li et al. improved PrefixSpan algorithm and proposed an improved sequential pattern mining (ISPM) algorithm. This algorithm can significantly reduce the construction times of the projection database, thus improving the efficiency of sequential pattern mining, The mining results are reordered according to the value of sequence patterns to find the most basic sequence patterns [5]. Shen et al. discussed the optimal time and threshold of homocysteine (Hcy) detection, providing a basis for early clinical prevention of PIH [6].

However, it is difficult to set the support threshold of the SPADE algorithm. Because the results of frequent sequence mining are highly dependent on support, when more minor support is used, a large number of periodic redundant sequences may be generated. In contrast, a more extensive support threshold is used, fewer frequent sequences may occur, and some vital information may be lost. Hu et al. proposed a pattern mining algorithm based on multiple support degrees to solve this problem. Amphawan proposed Top-K frequent pattern mining. Ruiyang et al. introduced logic theory into pattern mining algorithms to optimize the support threshold. However, it is challenging to implement the above methods in practical application. This article adopts statistical ideas, uses the relationship between the support threshold and the number of frequent sequences, considers the characteristics of the medical data in the electronic medical record and the drug data of hypertensive patients, and proposes an improved SPADE algorithm to solve the problem that the threshold of support is difficult to set.

A sequence pattern mining algorithm was used to study the drug sequence of hypertensive patients. Then, it was applied to obstetric hypertension patients, and the clinical efficacy of drugs was analyzed.

The specific pathogenesis of pregnancy hypertension syndrome has been studied continuously. Hypertension during pregnancy may be the first sign of preexisting pathological changes that can lead to adverse maternal, fetal, and neonatal outcomes. Early resolution of the hypertensive disease may not change the course or proficiency of the disease. Still, prompt detection and treatment can prevent not only hypertensive crisis but also alter adverse fetal outcomes. Early cataloguing plays a crucial role in predicting pregnancy outcomes for both mother and baby. Platelet index is related to platelet functional status and is a new risk marker for detecting impending adverse effects of pregnancy hypertension syndrome [7]. OU equal-length non-coding RNA MALAT1 promotes the development of gestational hypertension by regulating the miR-150 ‐5p/ET‐1 axis to enhance oxidative stress and inflammation [8]. Low vitamin D intake should be considered as a possible risk factor for PIH [9]. Li et al. conducted a nested case-control study to examine the relationship between circulating SFA and risk of PIH [10]. Yozuka et al. assessed the relationship between total IgE levels in early pregnancy and the occurrence of gestational hypertension syndrome (PIH) in a large Japanese cohort [11].

A sequence pattern mining algorithm was applied to the medication of pregnant hypertensive patients. The results showed that the 16% total treatment was about 96.6%, compared with the control group, suggesting a significant difference (*P* < 0.05). Comparison of blood pressure levels between the two groups also offered a better outcome (*P* < 0.05) and a substantial reduction of postpartum bleeding rates and perinatal complications in the observation group (*P* < 0.05). By studying the order of taking medications for hypertensive patients and combining various physical indicators of the patients, we can get the rule of taking medicines for hypertensive patients and make recommendations. It was applied to obstetric hypertension patients to analyze the clinical efficacy of drugs.

## 2. Research Methods

### 2.1. Sequential Pattern Algorithm

The improved SAPDE algorithm is adopted. Firstly, a mapping relation *f* is defined, and the mapping relation is composed of the number of frequent sequences *m*, and the support threshold min_sup is *m* = *f*(min_sup). A small support threshold is selected as the initial value, and then the support threshold increases linearly; *m* values are calculated under different min_sup, respectively. When *m* encounters the extreme point for the first time, the corresponding min_sup is the optimal support threshold. The obtained min_sup value is taken as the support threshold of the SPADE algorithm, and the SPADE algorithm is executed.

### 2.2. Drug Therapy

Fifty-eight pregnancy-induced hypertension patients were randomly selected as the subjects of this study and grouped for treatment. All the parturients were diagnosed with pregnancy-induced hypertension syndrome by clinical examination. All of them had no severe dysfunction of other vital organs, no adverse reactions to the drugs used in this study, and all were single pregnancy. They knew the purpose and method of this study and volunteered to participate. The control group was treated with nifedipine, and the observation group was treated with captopril. There were 29 cases in each group.

Control group: all patients received clinical examination after admission and received clinical treatment with nifedipine. Usage and dosage: the initial dose was 10 mg/time, twice a day, and the amount was adjusted once every three days according to the specific situation of the patient, but the maximum dose should not exceed 20 mg/time.

Observation group: based on the control group, captopril was added for clinical treatment. Usage and dosage: the initial dose is 6.25 mg/time, three times a day. Suppose the patient does not have obvious curative effects after treatment. In that case, the dosage should be adjusted appropriately, the control dose was 12.5 mg/day, and three months was taken as a treatment period for both groups. The therapeutic effects were compared after a treatment period.

### 2.3. Efficacy Evaluation Criteria

After treatment, the patient's blood pressure returned to normal, and clinically related symptoms disappeared, which can be judged as a significant effect. After treatment, patients' blood pressure is reduced by more than 10 mmHg compared with before treatment, and the clinical symptoms are significantly improved. No significant difference in the condition of patients before and after treatment is considered invalid. Apparent efficiency + efficiency = total efficiency.

### 2.4. Statistical Treatment

SPSS17.0 statistical software was used to process the data. The enumeration data were represented as %, *χ*2 test was used, the measurement data were defined as mean ± standard deviation, and *t*-test was used. If *P* < 0.05, it was proved to be statistically significant.

### 2.5. Generation of Sequence Rules

When generating sequence rules with frequent sequences, the last item of the sequence is the conclusion of the sequence rules, and all items in the sequence, except the last item, are the conditions for generating sequence rules. For special single frequency sequence, the null set is taken as the condition, and the 1-frequent sequence is taken as the conclusion to generate the rule. For example, the generation rule of single frequency sequence (< {thiazide diuretics} >) is (< {} > - < {thiazide diuretics} >), which indicates that doctors can prescribe thiazide diuretics according to their indicators in patients with hypertension for the first time.

## 3. Result Analysis and Discussion

### 3.1. Data Collection

A total of 913 records were selected from the medical record database of 528 hypertensive patients taking drugs, and each paper had four attributes, namely, medical record number, visit time, number of medications, and prescription drugs. The data are detailed in Table 1.

Due to the variety and complexity of drugs for treating hypertension, the sequence data are relatively sparse through the experiment. The scant data resulted in unsatisfactory mining results, so this paper classified hypertension drugs into 14 drug categories according to the hypertension prevention and treatment guidelines.

Drug products and drug categories are described in Table 2.

After classification and summary, the experimental dataset (MD) has four attribute values: the serial number of patients, the time of visit, the number of prescription drugs prescribed by doctors, and the type of drugs defined. The dataset is input into the sequence database, and the data format is shown in Table 3.

### 3.2. Judgment and Results of Support Threshold

MD was taken as a specific dataset to determine the support threshold, and a GSP algorithm was applied to obtain the determination results of the support threshold. The results are shown in Table 4.

As shown in Table 4, when min_ When sup = 0.001 is used as the initial value, the first extreme point appears. When min_sup = 0.007, M = 37, which is equal to the value of M. When min_sup = 0.008. Therefore, the optimal support threshold min_sup = 0.007 was finally obtained. It can also be intuitively reflected that when min_sup = 0.007, it is the optimal support threshold for this dataset, as shown in Figure 1.

MD was randomly divided into two datasets, MD1 and MD2. The GSP algorithm is applied, respectively, to obtain the results, as shown in Figure 2; when the MD dataset was reduced to half of the original value, MD1 showed the first extreme point when the *M* value appeared at min_sup = 0.006; for MD2, the first extreme point appeared when *M* was min_sup = 0.007. Then, MD was randomly divided into 4: MD3, MD4, MD5, and MD6, and the GSP algorithm was applied. It is found that the *m* value of these four datasets all appears at the first extreme point when min_sup = 0.007, as shown in Figure 3. For a particular dataset MD, if you only change the size of the dataset, the number of frequent sequences *M* appears at the first extreme point when the support threshold is min_sup = 0.007. Hence, the optimal support threshold is of dataset MD is verified again to be 0.007.

The average support reaches the extreme point for the first time at 0.007, min_sup = 0.007; when the average support = 0.018 and min_sup = 0.008, average support = 0.018, as shown in Figure 4. So, it is verified that min_sup = 0.007 is appropriate. At the same time, the average confidence also reaches the first extreme point at 0.007, and when min_sup = 0.007, the average confidence is 0.1712.

### 3.3. Mining Frequent Sequences

min_sup is set to 0.007 as a parameter. The sequential pattern mining algorithm continues to be executed to obtain the frequent sequence set *F*. There are 37 regular sequences in set F, and some periodic sequences and their support degrees are listed in Table 5.

### 3.4. Generation of Sequence Rules

Generating Sequence Rules with Frequent Sequences Here, the last item of the sequence is taken as the rule's conclusion, and all the items except the last item in the sequence are taken as the condition of the rule to generate sequence rules. For special 1-frequent sequences, the null set is taken as the condition, and the 1-frequent sequence is taken as the conclusion to generate the rule. For example, the 1-frequent sequence (<{thiazide diuretic} >), the rule generated by it is (<{} > - > < {thiazide diuretic} >), which indicates that patients diagnosed with hypertension for the first time, a doctor may prescribe a thiazide diuretic based on its indicators.

When generating sequence rules, the minimum confidence of 0.01 was selected, and a total of 37 sequence rules were generated from frequent sequences. Some sequence rules are listed in Table 6, where < {Beta blocker}≥> <{ACEI, Thiazide diuretics, beta blockers}>, indicating that the patient was on a previous beta blocker, and the last medication was insufficient to control blood pressure due to the progression of the disease. Doctors may prescribe ACEI, thiazide diuretics, and beta-blockers, which is a combination of three drugs.

### 3.5. Visualization of Rules

The mined rules are visualized below, and the sequence rule diagram is shown in Figure 5.

The sequence rules of medication for hypertensive patients combined with various physical indicators of the patients were used for obstetric hypertension patients.

### 3.6. Comparative Analysis of Clinical Data between Two Groups of Patients with Different Medications

The total effective rate in the observation group was 96.6%, and that in the control group was 79.3%. The data comparison between the two groups indicated *P* < 0.05, showing statistical significance in Table 7.

After treatment, the diastolic blood pressure and systolic blood pressure levels of the two groups were compared. The results showed that the observation group was significantly better than the control group (*P* < 0.05), as shown in Table 8.

The rate of postpartum haemorrhage and the incidence of perinatal complications were compared between the two groups. The results showed that the observation group was significantly lower than the control group (*P* < 0.05), in which 3 cases of premature delivery occurred in the control group, there were 2 cases of neonatal asphyxia, 2 cases of placental abruption, and 1 case of placental distress. Preterm labour and placental abruption occurred in 1 point in the observation group (see Table 9).

## 4. Conclusions

An improved SPADE algorithm is proposed to solve the problem that the support threshold of the SPADE algorithm is difficult to set. According to the relationship between the support threshold and the number of frequent sequences, the support threshold corresponding to the first extreme point on the change curve was selected as the optimal support threshold. Applying the improved SPADE algorithm to the sequence data of hypertension patients taking a medication history, mining frequent sequence patterns, and then converting regular sequence patterns into sequence rules can guide drug therapy step by step.

However, the SPADE algorithm is difficult to set. Since frequent sequence mining is very dependent on the support, a large number of frequent redundant sequences may appear when using a remote mount. However, using a large support threshold may produce fewer frequent sequences and may lose some important information. The specific pathogenesis of pregnancy hypertension syndrome has been continuously studied. Pregnancy hypertension may be the first sign of having pathological changes first, leading to adverse maternal, fetal, and neonatal outcomes. Early resolution of hypertension may not alter the progression and proficiency of the disease.

Nevertheless, timely detection and treatment can not only prevent the risk of hypertension but also change the adverse fetal outcome. The sequence rules of medication for hypertensive patients were combined with the patients' physical indicators for a recommendation. For patients with obstetric hypertension, a combination of nifedipine and captopril is recommended. Through the comparison of the observation group and control group, we study the curative effect of various drugs. The results showed that the total effective rate of the observation group was about 96.6%; compared with the control group, the result indicated that the difference was significant (*P* < 0.05). The comparison of blood pressure levels between the two groups after treatment also showed that the results of the observation group were ideal (*P* < 0.05). In addition, the incidence of postpartum haemorrhage and perinatal complications in the observation group was also significantly reduced (*P* < 0.05). Therefore, the combination of medication for pregnancy hypertension syndrome can effectively improve the treatment effect of the disease and reduce the rate of postpartum haemorrhage and the incidence of perinatal complications.

## Figures and Tables

**Figure 1:** Relationship between min_sup and M of dataset MD.

**Figure 2:** Relationship between min_sup and m of datasets MD1 and MD2.

**Figure 3:** Relationship between min_sup and m of datasets MD3, MD4, MD5, and MD6.

**Figure 4:** Validation of optimal support threshold.

**Figure 5:** Sequence rules.

**Table 1:** Dataset description.

Medical record no.	Number of drugs	Prescription drugs
000071	1	Nifedipine
011224	1	Silas split
001113	1	Silas split
000137	2	Cilapril hydrochlorothiazide

**Table 2:** Description of hypertensive drugs and drug categories.

Prescription drugs	Drug category
Amlodipine	Dihydropyridines CCB
Diltiazem sustained-release tablets	Non-dihydropyridines
Ogilvy sha Tanzania	ARB
Indapamide	Thiazide diuretics
Captopril	ACEI
Yipuliton	Aldosterone antagonist
Metoprolol	*β* beta-blockers
Labetalol	*α*-*β* beta-blockers

**Table 3:** Input data format description.

Sid	Count	Items
1	1	Dihydropyridines CCB
2	1	ACEI
3	1	ACEI
4	2	ACEI thiazide diuretics
4	2	ACEI *β* beta-blockers

**Table 4:** Judgment results of the support threshold value.

min_sup	m/time	min_sup	m/time
0.001	584	0.006	44
0.002	115	0.007	37
0.003	90	0.008	37
0.004	65	0.009	32
0.005	58	0.010	32

**Table 5:** Frequent sequence.

The sequence	Support
<{ACEI}>	0.4166
<{ACEI thiazide diuretics}>	0.2309
<{*β* Beta-blockers}>	0.1284
<{ACEI dihydropyridines CCB thiazide diuretics}>	0.1076
<{*β* beta-blockers},{ACEI *β* beta-blockers}>	0.0277
<{ARB},{*β* beta-blockers ARB}>	0.0053
…	…

**Table 6:** Sequence rule description.

The rules	Support	Degree of confidence	Ascension degree
{}=> {thiazide diuretics}	0.0481	0.0481	1
{}=> {ACEI *β* beta-blockers}	0.0503	0.0503	1
{}=> {ACEI thiazide diuretics *β* beta-blockers}	0.0646	0.0646	1
{*β* beta-blockers}= > {ACEI *β* beta-blockers}	0.0278	0.2162	2.71
<{*β* beta-blockers}, {ACEI thiazide diuretics}≥> <{ACEI thiazide diuretics *β* Beta-blockers}>	0.0122	0.7	6.83
<{*β* beta-blockers}> = > <{ACEI thiazide diuretics *β* beta-blockers}>	0.0243	0.1891	1.84

**Table 7:** Comparative analysis of the total effective rate of clinical treatment between the two groups.

Group	The number of cases	Excellent	Useful	Invalid	Total effective rate (%)
Control group	29	13	10	6	23 (79.3)
Observation group	29	16	12	1	28 (96.6)
*χ*2	—	—	—	—	4.500
*P*	—	—	—	—	<0.05

**Table 8:** Comparison of blood pressure levels between the two groups after treatment.

Group	The number of cases	Diastolic blood pressure (mmHg)	Systolic blood pressure (mmHg)
Control group	29	94.4 ± 6.7	131.5 ± 7.4
Observation group	29	81.1 ± 4.3	116.3 ± 5.8
*χ*2	—	8.996	8.705
*P*	—	<0.05	<0.05

**Table 9:** Comparison of postpartum bleeding rate and perinatal complication rate between the two groups.

Group	The number of cases	Two months after surgery	Six months after surgery
Control group	25	47.36 ± 9.26	89.63 ± 10.25
Observation group	25	16.32 ± 3.52	43.65 ± 11.42
*χ* ^2^	—	12.052	11.242
*P*	—	0.000	0.000

## Data Availability

The data used to support the findings of this study are available from the corresponding author upon request.
